This article has been retracted.

# Epoxy Resins Toughened with Surface Modified Epoxidized Natural Rubber Fibers by One-Step Electrospinning

**DOI:** 10.3390/ma10050464

**Published:** 2017-04-27

**Authors:** Joo Ran Kim, Jung J. Kim

**Affiliations:** 1 Fiber Science, Cornell University, Ithaca, NY 14853, USA; jk992@cornell.edu; 2 Department of Civil Engineering, Kyungnam University, Changwon-si 51767, Korea

**Keywords:** natural rubber fibers, epoxy resin, toughening, surface modification

## Abstract

Epoxidized natural rubber fibers (ERFs) are developed through one-step electrospinning and directly deposited into epoxy resins without collecting and distributing of fibers. The shape of ERFs shows rough surface due to different evaporation rate of solvent mixture consisting of chloroform and dichloromethane and the average diameter of ERFs is 6.2 µm. The increase of ERFs loading from 0 to 20 wt % into the epoxy resin increases the fracture strain significantly from 1.2% to 13% and toughness from 0.3 MPa to 1.9 MPa by a factor of 7. However, the tensile strength and Young’s modulus decrease about 34% from 58 MPa to 34 MPa and from 1.4 GPa to 0.9 GPa, respectively. Due to the crosslinking reactions between oxirane groups of ERFs and amine groups in the resin, surface roughness and the high aspect ratio of ERFs, ERFs result in more effective toughening effect with the minimum loss of tensile properties in epoxy resins.

## 1. Introduction

Electrospinning as an efficient and versatile technology has been developed for generating ultrafine fibers in a variety of materials, such as polymers, inorganic materials, and hybrid materials [1]. These fibers or non-woven fibrous membranes exhibit diameters ranging from a few nanometers to a few micrometers and have advantages of large surface area-to-volume ratios and various morphological modifications [2]. Electrospinning system typically consists of three basic components: a high voltage supply, a Taylor cone and a metal collector [3]. The electrodes contain a high voltage supply, with one connected to the polymer solution being metered and the other connected to the collector. As electrostatic repulsion counteracts the surface tension on the Taylor cone, the polymer solution is stretched to draw threads [4]. This stretched polymer solution evaporates the solvent to form solid fibers before fibers reach to the collector [5]. During electrospinning, the morphology or mechanical properties can be easily modified by tuning many parameters such as polymer concentration, distance between a Taylor cone and a collector, applied voltage, syringe feeding rate, etc. depending on applications such as biomaterials, reinforcement, barrier textiles and toughening [6,7,8,9]. Among these applications, brittle thermoset resins have been studied to increase the material toughness using electrospinning technique [7]. Epoxy resins toughened with electrospun polysulfone nanofibers showed an increase in fracture toughness (*G*_IC_) of 158%, 261% and 281% at 1, 3 and 5 wt % of fiber loadings, respectively [10]. The epoxy reinforced with carbon fibers composite showed 100% improvement in fracture toughness as 20% polycaprolactone nanofiber was incorporated into the epoxy composites to increase the interlaminar fracture toughness [11]. Electrospun poly(vinyl pyrrolidone)/tetraethyl orthosilicate/silica nanoparticle nanofibers (2% loading) improved the fracture toughness by 1.9 times that of neat polypropylene resin [12]. Nanofibers composed of styrene-butadiene-styrene (SBS) block copolymer as a rubbery core and polyacrylonitrile (PAN) as a hard sheath have been produced via coaxial electrospinning, and can be used to improve the toughness of epoxy matrix increased impact energy up to 150% [13]. 

Many studies have investigated improving toughness of epoxy resin using synthetic copolymers and metal derivatives as toughening agents such as carboxyl-terminated acrylonitrile butadiene, synthetic ductile polymers such as the acrylic rubber, hydroxy-terminated butadiene or acrylonitrile butadiene, epoxy-terminated acrylonitrile butadiensbse, epoxy-terminated butadiene and amine-terminated acrylonitrile butadiene [14,15,16,17]. 

However, little research has been conducted on eco-friendly toughening agents to improve brittle epoxy resins. For example, epoxy resins with 60% functionalized green halloysite nanotubes resulted in increased impact strength to about 5.8 kJ m^−2^, 1.5 times that of neat epoxy resin even metal conductivity of 0.85 W m^−1^ K^−1^ [18]. After adding 10% hyperbranched polyurethane into epoxy resins, the impact strength was increased to triple the amount of neat epoxy [19]. In another example, silicone skeleton was used as a toughening agent added into the epoxy resin, showing increased impact, flexural and tensile strength of epoxy resin by about 92.5%, 36.0% and 88.6%, respectively, compared to neat epoxy resin [20].

The problem in ductile toughening agents is that most resins experience a decline in their tensile properties with the addition of ductile materials. Hence, good interfacial bonding via chemical reactions between the matrix and the toughening agent has been an active research area in order to improve the toughness without loss of tensile properties in the matrix. For example, as 0.5 wt % dodecane functionalized tannic acid incorporated into epoxy resin as the toughening agent increased the impact strength by up to 196% compared to that of neat epoxy [21]. This tendency was due to good interfacial bonding between terminal hydroxyl groups of dodecane functionalized tannic acid and the epoxy matrix [21]. Glycerol (10 wt %) was used to improve toughness of poly(lactic acid) (PLA) matrix, resulting in strain at break of up to 93% and fracture stress of 48 MPa compared to neat PLA matrix with strain at break of 2.3% and fracture stress of 64 MPa. Again, this trend is due to esterification reaction occurring at the interface between the hydroxyl groups of glycerol and the carboxylic groups of PLA [22]. Eco-friendly natural toughening agents such as epoxidized natural rubber (ENR) and liquid natural rubber have been found to be effective in improving the toughness in brittle resins because of functional groups such as oxirane groups or hydroxyl groups [23,24,25]. One explanation is that the oxirane groups of ENR are able to react with carboxyl, amine, glycidyl and hydroxyl groups of matrices, crosslinking with ENR to offer good interfacial bonding in the matrix [26]. One example is biodegradable PLA matrix and ENR blend via chemical reactions between oxirane groups and carboxylic groups, resulting in improved toughness and tensile properties [27,28].

The primary objectives of this study were to develop micro-sized green elastic ENR fibers (ERFs) with surface modification through one-step electrospinning. Figure 1 shows the one-step electrospinning system developed in this study for the ERFs production and concurrently distribution of ERFs with epoxy resin. ERF loading was varied at 5, 10, 15 and 20 wt % into epoxy resins (E-ERF 5, E-ERF 10, E-ERF 15 and E-ERF 20, respectively) and its effect on toughness and other mechanical properties was analyzed.

## 2. Results and Discussion

Figure 2 shows the morphology of ERFs produced using 1% ENR polymer concentration. The range of diameter of ERFs varied from 1.6 µm to 13 µm and the average diameter of ERFs is about 6.2 µm as shown in Figure 2a. The surface of ERFs displays bumpy (spines-like) and rough edges as shown in Figure 2b. This morphology is related to a rapid evaporation of the solvent while the fibrous jet is accelerated to the metal collector. Megelski et al. [29] have studied the effect of different solvents such as acetone, chloroform, tetrahydrofuran and their mixtures on the morphology of fibers. When polyethylene glycol (PEO) was spun from chloroform displayed rougher surface of fibers than other fibers used other solvents [29]. Similar studies showed that the boiling temperature of solvent was associated with surface roughness and diameter size [30]. Electrospun fibers showed an increase in surface roughness and pores with increasing boiling point of the solvent mixture since the boiling temperature is related to volatility of solvents [30]. As ENR is dissolved in only dichloromethane while keeping other parameters constant, ERFs display smooth surface. As the mixture of chloroform and dichloromethane was used as the solvent for ENR, the mixture of solvents influences the surface roughness in this study. Since ERFs are directly deposited into epoxy resins heated at 40 °C during electrospinning, the mixture of two solvents has different boiling temperature (*T_b_*) and volatility rate because chloroform (*T_b_*: 61 °C) has higher boiling temperature than dichloromethane (*T_b_*: 39 °C) [29]. 

The internal structures of ERFs are shown in Figure 3. Left images are all brightfield images, whereas right images are fluorescent images that indicate the presence of ENR stained with a fluorescent dye, appearing green colored. The ERFs produced using 1% polymer concentration have long rod, non-porous, and rough surface, as shown in Figure 3a,c. A close examination of the white square area in Figure 3a,b demonstrates the rough surface at the edges of the ERFs. Their green color indicates that the ERFs are composed of ENR and have rough edges as shown in Figure 3b,d. The weak green signal indicates ERFs have smaller diameter or thinner region of ENR (less ENR concentration); however, the strong green signal indicates larger diameter or thicker area of ERFs. The results from a Confocal laser scanning microscopy (CLSM) images confirm the morphology of ERFs as shown in SEM results in Figure 2. 

Figure 4 shows attenuated total reflection Fourier transform infrared spectroscopy (ATR-FTIR) spectra of neat ERFs, neat epoxy and all E-ERF resins. Neat epoxy specimen shows transmittance peaks at 860 cm^−1^ (epoxy C–O–C ring deformation) [31], 1020–1250 cm^−1^ range (C–N stretching), 1375 cm^−1^ and 1494 cm^−1^ (CH and CH_2_ deformation), 1528 cm^−1^ (NH stretching) and 2862–2937 cm^−1^ range (CH and CH_3_ asymmetric stretching) [32]. The broad peak around 1600 cm^−1^ corresponds to NH_2_ bending of excess amine group from the curing agent in the epoxy resin. Neat ERFs transmittance peaks at 751 cm^−1^, 852 cm^−1^ and 1246 cm^−1^ corresponding to the oxirane groups appeared in the spectra [24]. 

The E-ERF resins show additional peak at 3000–3600 cm^−1^ range to indicate the presence of hydroxyl groups (–OH) produced by crosslinking reaction between oxirane groups of epoxy resin or ENFs and amine of the curing agent, as shown in Figure 4b. The oxirane group is shown to open up during curing process and the reaction product is secondary amines with hydroxyl groups [33]. Two hydroxyl groups of secondary amines can react further to form ether linkages [33]. In Figure 4a, the reaction between oxirane groups of ERFs or epoxy resin and excess amine of the curing agent shows peak at 1020–1250 cm^−1^ range corresponding to C–N linkages [34]. The increase of ERFs loading into epoxy resin shows increase in peaks of C–N (1020–1250 cm^−1^ range), C–O–C (ether stretching vibration at 945 cm^−1^) and –OH (3000–3600 cm^−1^), as shown in Figure 4a. The increased transmittance peaks demonstrate that E-ERF resins show additional crosslinking reactions between oxirane group of ERFs and excess amine or hydroxyl group in epoxy resins [35].

Figure 5 presents differential scanning calorimetry (DSC) thermograms of neat epoxy, neat ERFs, and all E-ERF resins at different loading of ERFs scanned from −50 to 200 °C. In the present study, neat ERFs show *T*_g1_ (glass transition temperature of ENR) at −25 °C, whereas neat epoxy matrix shows *T*_g2_ (glass transition temperature of epoxy resin) at 55 °C. E-ERF resins, however, show little change in *T*_g1_ from −28 to −25 °C but significant change in *T*_g2_ from 55 to 65 °C as ERFs loading increases from 0 to 20 wt %. At 5 wt % loading of ERFs in epoxy resin, there is little increase in *T*_g2_. However, with the 10% addition of ERFs, *T*_g2_ increases by 7 °C. This increasing trend continues with ERFs loading of 15 and 20 wt % in epoxy resins to 63 and 65 °C, respectively. This trend is attributed to cross-linking reactions between oxirane group of ERFs and excess amine or hydroxyl group in epoxy resins to create a 3D cross-linking structure. These cross-links increase the chain length and interactions between chains, resulting in limited freedom to rotate about the bonds and consequently, increases the *T*_g2_ temperature of E-ERF resins [36,37]. The finding is in line with the observations made by Thomas et al. [38] for epoxy resin toughened with liquid natural rubber. Other researchers showed this shift of *T*_g_ with increasing loading concentrations of liquid rubber [39]. They explained that the addition of liquid natural rubber into the epoxy resin increased the curing temperature by allowing crosslinking reactions to occur between the epoxy resin and hydroxyl or carboxylic groups of rubber [40]. 

Figure 6 presents dynamic mechanical analysis (DMA) plots of E-ERF resins scanned from −50 to 100 °C. The storage modulus (*E*′) of E-ERF resins is plotted as a function of temperature in Figure 6a. The storage modulus of neat epoxy resin shows nearly 5 GPa, whereas E-ERF resins display around 4.5 GPa. In the case of E-ERF resins, as the temperature increases, there is a sharp decrease in storage modulus starting around −28 °C, corresponding to *T*_g1_ of ENR. The *E*′ for neat ENR resin shows the final storage modulus close to 0 MPa at 60 °C, whereas E-ERF resins show *E*′ values above 4 GPa at 60 °C. 

The mechanical loss factor (tan *δ*) plots for E-ERF resins are shown in Figure 6b. The intermolecular interactions between ENR and epoxy resin brought about different altering trends of *T*_g_ because ENR is at elastic state whereas rigid epoxy resin stays at glassy state. The tan *δ* peak at around −25 °C represents relaxation of the neat ENR. As ERFs loading increases from 0 to 20 wt %, the *T*_g1_ values of E-ERF resins decrease slightly from −28 to −25 °C; however, *T*_g2_ values of E-ERF resins increase from 51 to 65 °C. The reason is that the chemical crosslinking reactions between oxirane groups of ENR and excess crosslinking agent in epoxy resin occur and result in long molecular chain and offer higher than intermolecular hydrogen bonding. Therefore, free motion of epoxy molecular chain segments are restrained, which results in an increase of *T*_g2_ [41,42]. 

Figure 7 shows the tensile fracture surfaces of E-ERF 10 resins. For neat epoxy resin, many layered structures or sharp cracks can be seen in Figure 7a. Many studies have reported this appearance to be the distinctive brittle fracture surface of thermoset resins [43,44]. However, after adding ERFs to epoxy resins, the resins decrease in brittle features and sharp crests on the fracture surfaces. As the loading of ERFs added into epoxy resins increase, the fracture surfaces display rougher and glossier features without the formation of cracks along the fiber direction which indicates the primary characteristic of weak interfacial bonding between fibers and resins [45]. Figure 7b shows the tensile fracture surface of E-ERF 10 resin, clearly demonstrating that ERFs are seen protruding long fibers from the epoxy resin. The ERFs show good dispersion with the wide range of diameter sizes in in E-ERF 10 resin. The interface between ERFs and epoxy resin displays little fiber pullout, delamination or interface failure induced from weak interfacial bonding between fibers and resins. The strong interfacial bonding occurs by means of crosslinking reaction between oxirane groups of ERFs and amine groups of excess curing agent, increasing the load transfer of ERFs to the epoxy resin. Chemical reactions such as epoxy-amine reaction in the interface play a critical role for interfacial adhesion, specifically the oxirane group opening in the interface and the formation of covalent bonds with ERFs [46]. Figure 7c shows the top surface of the E-ERF 10 resin. ERFs display circular or entangled fibers on the surface; however, they still maintain their rough surface to help ERFs to bond physically to epoxy resin, as shown in Figure 7d. Figure 7e shows the bridging zone of the E-ERF 10 resin. It demonstrates an effective toughening mechanism through the addition of ductile materials such as rubber materials. ERFs effectively connect or bridge two fracture surfaces of the E-ERF 10 resins. Because of inherent toughness and high aspect ratio of ERFs, cracks larger than 500 µm are stopped from propagating into larger cracks. These results show that the adhesion between the ERFs and the epoxy resin are reasonably strong with the absence of breakage or pullout features [47]. The enlarged image (Figure 7f) shows the nanoweb (fishnet-like) formation in the bridging zone. These nanoweb formations have been explained by Liu et al. [48]. The solvent remained in electrospun fibers caused by the incomplete solvent evaporation led to form the connected fibers or nanoweb [48,49]. 

After curing, neat epoxy resin and all E-ERF resins are tested for their tensile properties. Figure 8 shows typical tensile stress–strain plots of neat epoxy resin and all E-ERF resins and their tensile properties are summarized in Table 1. The increase in ERFs loading in the epoxy resin from 0 to 20 wt % increase the fracture strain significantly from 1.2% to 12.8% and the toughness at break increase seven times from 0.3 to 1.9 MPa. Remarkably, the tensile strength and Young’s modulus show only a minimal decline of 34% from 58 to 34 MPa and from 1.4 GPa to 0.9 GPa, respectively. The neat epoxy specimens are broken in a brittle manner with no apparent yielding, revealing the typical characteristic of a thermoset resin. The tensile strength decreases with an increase in ERFs loading since the ERFs act as stress concentrators, causing a decrease in facture strength and Young’s modulus [50]. E-ERF 5 and E-ERF 10 show about 1.2 GPa and 1.1 GPa of modulus, and 52 MPa and 47 MPa of fracture strength, respectively, compared to that of neat epoxy resin having modulus of 1.4 GPa and tensile strength of 58 MPa. Compared to other studies, epoxy resin containing ENR particles (not in fiber form) showed much loss in tensile properties [24,51,52]. For example, epoxy resin with 12% liquid epoxidized natural rubber (particle size 0.48 to 0.67 in diameter) increased 125% impact toughness, but decreased tensile properties by 15 MPa from 65 MPa to 50 MPa, compared to neat epoxy resin [51]. As 20% ENR was added into epoxy resin it have been reported to improve the impact strength of 2.55 J m^−1^ and *K*_IC_ value of 1.79 MPa m^1/2^ but the modulus decreased to half that of neat epoxy resin [52]. However, the fiber form of ERFs results in significantly higher strain, fracture toughness, and minimal loss of tensile properties when incorporated into the epoxy resin in this study. High aspect ratio due to its fiber form contributes to better interfacial interaction, flexibility in surface functionalities, and superior mechanical performance than the particle form of ENR [53]. The minimal loss in strength and modulus can be explained by the crosslinking reactions between oxirane groups and amine which result in a very effective 3D structure that helps to maintain the tensile properties. 

## 3. Experimental Section

### 3.1. Materials

Araldite^®^ GY 6010 (MW: 11,000–14,000, unmodified DGEBA liquid) was purchased from Huntsman Co. (Salt Lake City, UT, USA). Aradur^®^ 956-2 (modified aliphatic amines) was purchased from Krayden Inc. (Denver, CO, USA). Epoxidized natural rubber (ENR, 50 mol % conversion) was donated by Malaysian Rubber Board. Adirondack green 520 fluorescent dye, chloroform, dichloromethane were purchased from Sigma Aldrich Chemical Co. (St. Louis, MO, USA).

### 3.2. Electrospinning of ENR Fibers

ENR (1 wt %) was dissolved in the mixture of 1:2 (*v*/*v*) of dichloromethane and chloroform and then stirred for 12 h at room temperature (RT). The solution was put into a 10 mL syringe, and electrospun into fibers (ERFs) with a high voltage of 12 kV. The syringe feeding rate used was 30 µL min^−1^ and the distance between the syringe needle tip (diameter: 1 mm) and the collector was 15 cm. Precured epoxy resin was placed above the bath containing metal collector and heated to 40 °C with stirred at 50 rpm. ERFs were directly deposited into the epoxy resin. 

### 3.3. Fabrication Process of Epoxy Composites at Different Loadings of ERFs

The curing agent, 35 wt % Aradur^®^ 956-2, was added into neat epoxy matrix (DGEBA) and stirred at 50 rpm for 30 min. Electrospun ERFs using 1 wt % ENR polymer concentration were directly deposited into the epoxy resin. Then the epoxy resin containing ERFs at different loadings was poured into a Teflon^®^ mold (127 × 127 mm) and precured for 3 h at 40 °C. The epoxy matrix containing ERFs was cast in the form of sheets and the epoxy sheets were then cured in the oven at 1 h for 100 °C. Afterwards, all specimens were conditioned at 21 °C and 65% RH for 72 h prior to their characterization.

### 3.4. Thermal Analysis

All epoxy resins containing ERFs at 5, 10, 15 and 20 wt % (E-ERF 5, E-ERF 10, E-ERF 15, and E-ERF 20, respectively) were tested their thermal properties. E-ERF resins were scanned on differential scanning calorimeter (TA-DSC 2000, TA instruments Inc., New Castle, DE, USA) at a heating rate of 5 °C min^−1^ from −50 to 200 °C to evaluate the changes in their thermal properties under a nitrogen flow rate of 100 mL min^−1^.

### 3.5. Tensile Properties of E-ERF Resins

All E-ERF resins were cut by a laser cutter to obtain the dimensions of 50 mm × 10 mm and were characterized for their tensile properties according to ASTM D882-02 standard at a strain rate of 0.6 mm min^−1^ and gauge length of 30 mm. All tests were performed on Instron universal tensile tester (Instron, Model 5566, Instron Co., Canton, MA, USA) using at least ten specimens [54].

### 3.6. Dynamic Mechanical Analysis of E-ERF Resins

Dynamic mechanical properties of E-ERF resins were analyzed using DMA (DMA Q800, TA Instruments, New Castle, DE, USA) in 3-point bending mode. Resins were cut into the final specimen dimensions of 30 mm × 10 mm and scanned from −50 to 100 °C at a ramp rate of 5 °C min^−1^. All tests were performed at 5 µm amplitude and sinusoidal tensile stress (frequency, 1 Hz), and conducted at least three times [55]. 

### 3.7. Morphological and Chemical Analyses

Microstructures of the tensile fracture surfaces of all E-ERF resins were analyzed using Tescan Mira3 FESEM. ATR-FTIR (Magna 560, Nicolet Instrument Technologies, Fitchburg, WI, USA) was used to confirm crosslinking reactions of E-ERF resins. Neat ENR, neat epoxy matrix and all E-ERF resins were scanned from 700 to 4000 cm^−1^ wavenumbers with a total of 300 scans and a resolution of 2 cm^−1^. ENR solution was stained with 0.5% Adirondack green 520 fluorescent dye of ENR before electrospinning. Then, it was electrospun directly into epoxy matrix. The resins were analyzed using a confocal laser scanning microscope (CLSM; Zeiss LSM710, Thornwood, NY, USA) and 520 nm excitation filter with 25× objective lens.

## 4. Conclusions

A convenient one-step electrospinning was developed for green elastic natural rubber fibers. ERFs were directly deposited to epoxy resins without collecting or redepositing of fibers. The surface of ERFs displayed bumpy (spines-like) and rough edges due to different volatility rate of solvents. The range of diameter of ERFs varied from 1.6 µm to 13 µm and the average diameter was approximately 6.2 µm. The increase of ERFs loading from 0 to 20 wt % into epoxy resins increased the fracture strain significantly from 1.2% to 12.8% and toughness at break from 0.3 MPa to 1.9 MPa, an increase by a factor of 7. However, Young’s modulus decreased minimally from 1.4 GPa to 0.9 GPa. E-ERF resins showed the presence of strong interfacial bonding between the ERFs and the epoxy resin without breakage or pullout of fibers. Inherent rubber toughness and high aspect ratio of fiber form of ERFs could contribute to efficient energy dissipation, since effective crosslinking reactions between the oxirane groups and amine or hydroxyl groups in epoxy resin allow the 3D structure to serve as an effective toughening agent. Green elastic ERFs could be useful in many applications such as construction materials, biomaterials, smart textiles, automotive and aerospace, therefore replacing petroleum-derived elastic fibers.

## Figures and Tables

**Figure 1:** One-step electrospinning to prepare ERFs into epoxy resins.

**Figure 2:** The morphology of micro-sized ERFs produced using 1% ENR polymer concentration.

**Figure 3:** The internal structures of micro-sized ERFs produced using 1% ENR concentration by CLSM: (**a**) the brightfield image of ERFs; (**b**) the fluorescent image of ERFs at low magnification; (**c**) the brightfield image of the white square area; (**d**) the fluorescent image of the white square area (green color corresponds to ENR stained with fluorescent dye).

**Figure 4:** (**a**) ATR-FTIR spectra of neat epoxy resin, neat ERFs and all E-ERF resins; (**b**) possible reactions between oxirane group and amine to form the secondary amines with hydroxyl groups and two secondary amines form ether linkages in epoxy resin.

**Figure 5:** DSC thermograms of neat ERFs, neat epoxy and all E-ERF resins.

**Figure 6:** DMA plots of neat epoxy resin, neat ENR sheet, and E-ERF resins at different loading of ERFs in the temperature range of −50 to 100 °C: (**a**) the storage modulus; and (**b**) the tan *δ* curves.

**Figure 7:** SEM images of fracture surface in tensile mode: (**a**) the fracture surface of neat epoxy resin; (**b**) the fracture surface of E-ERF 10 resins; (**c**,**d**) the top surface of E-ERF 10 resin; (**e**) bridging zone of E-ERF 10 resin; (**f**) nanoweb formation in bridging zone.

**Figure 8:** Typical stress–strain plot of neat epoxy resin and all E-ERF resins.

**Table 1:** Tensile properties of all E-ERF resins.

Type of Resins	Epoxy/ERF Composition (*w*/*w*)	Tensile Strength (MPa)	Tensile Strain (%)	Toughness at Break (MPa)	Young’s Modulus (GPa)
E-ERF	100/0	58 (1.6) *	1.2 (0.1)	0.3 (0.03)	1.4 (0.09)
	95/5	52 (1.2)	4.4 (0.3)	0.8 (0.1)	1.2 (0.05)
	90/10	47 (1.0)	7.5 (0.5)	1.4 (0.1)	1.1 (0.05)
	85/15	39 (0.8)	10.2 (0.4)	1.8 (0.2)	1.0 (0.04)
	80/20	34 (1.1)	12.8 (0.8)	1.9 (0.1)	0.9 (0.05)

* The values in parentheses are standard deviation.
